# Rule Extraction for Screening of COVID-19 Disease Using Granular Computing Approach

**DOI:** 10.1155/2022/8729749

**Published:** 2022-06-22

**Authors:** Seyyed Meysam Rozehkhani, Maryam Mohammadzad

**Affiliations:** Department of Computer Science, Faculty of Mathematics, Statistics and Computer Science, University of Tabriz, Tabriz, Iran

## Abstract

In the epidemic status of an unknown virus called Coronavirus, one of the main problems is inadequate access to treatment centers. Statistics show that many people are infected with the virus through unseasonable visits to medical centers immediately after noticing the initial symptoms similar to those reported for Coronavirus. Besides, unnecessary congestion at health centers reduces the quality of service to patients in urgent need of care. Since any external factor, including the virus, appears to have some symptoms after the onset of activity in the affected person, early diagnosis is possible. This paper presents an approach to classifying patients and diagnosing disease by symptoms, based on granular computing. One of the vital features of this method is the extraction of correct rules with zero entropy. This process is done based on a predefined classification of training datasets collected by experts. Granular computing has been a helpful approach in rule extraction and variety in recent years. Experimental results show that the proposed method can successfully detect COVID-19 disease according to its observed symptoms.

## 1. Introduction

By December 2019, 6 variants of Coronavirus were known to infect humans potentially. Four songs of the virus caused mild disease, and two, including SARS and MERS, were able to generate more severe disease [1]. Some vague reports of lung disease were reported in Wuhan, China, in late December 2019. Health researchers noticed the rapid transmission of the virus and took steps to manage the crisis. Coronavirus was the name given to this unknown virus by the World Health Organization on January 21, 2020. The number of people infected with the Coronavirus in 2020 exceeded the number of people infected with the SARS virus in 2002 [2]. According to recent global reports, the virus has now spread worldwide. The humanitarian costs of the Coronavirus outbreak continue to rise, with more than 452.394.748 people infected worldwide. The number of people who have died due to the virus has now exceeded 6.046.265 [3].

Coronaviruses range in size from about 60 nm to 140 nm in diameter. Under a microscope, a corona-like hyacinth appears on its surface, called the Coronavirus. The rate of transmission of the Coronavirus between humans is very high. When the virus enters a person's body, even long after recovery, that person's body is infected and can carry the virus. Ways of transmitting the virus include inhaling virus-infected droplets, touching virus-infected surfaces directly, and touching the mouth, nose, and eyes. The virus can also be transmitted through the feces of an infected person [4].

The emergence of uncertainty in detecting an unknown virus activity can be considered a challenge in computer science at this time. In the epidemic status of an unknown virus called Coronavirus, one of the main problems is inadequate access to treatment centers. Statistics show that many people are infected with the virus through unseasonable visits to medical centers immediately after noticing the initial symptoms similar to those reported for Coronavirus. Besides, unnecessary congestion at health centers reduces the quality of service to patients in urgent need of care. Since any external factor, including the virus, appears straight after the onset of activity in the affected person, early diagnosis is possible. This paper uses granular computing to classify patients based on their specific symptoms. Each person is regarded as an object that has attributes. These traits are the same symptoms identified in the patient. Granular computing can detect the presence or absence of disease using extracted rules. In the following, some introduction about Coronavirus and symptoms of COVID-19 diseases are provided.

### 1.1. Symptoms of COVID-19

Coronavirus causes a wide range of symptoms: fever and mild respiratory symptoms (upper respiratory tract infection), diarrhea, weakness, and lethargy. More severe symptoms contain progressive lung infection, respiratory failure, renal failure, and multiorgan failure. Just fever and just diarrhea are not common, but they are seen at the onset of the disease. The most common symptoms are fever and respiratory symptoms. Other laboratory symptoms like lymphopenia, thrombocytopenia, leukocytosis, elevated liver enzymes, and creatinine exist but may not have a good prognosis. The incubation period varies from 2 to 14 days. Coronaviruses usually have the highest rate of virus spread on day 4 of the illness, and then, the virus gradually reduces the burden on the body and transmits to others equally. It is possible to extend the disease to others for up to 24 hours after the end of fever and other symptoms [5]. 98% of patients with Coronavirus had a fever above 38°C, 76% had a cough, 44% had muscle fatigue and pain, and 55% had shortness of breath [6]. In [7], 1099 cases of COVID-19 disease were reported, in which a high percentage of fevers and dry coughs were reported. In this paper, symptoms such as diarrhea and vomiting are reported with a low percentage.

### 1.2. Prevention and Control of COVID-19 Infection

To limit the spread of the virus, the most significant step is to follow public health measures. A distance of 1.5 to 2 meters from each other and a ban on travel between different cities and no direct contact with infected people and people close to patients such as hospital staff are necessary to control the virus epidemic. The World Health Organization has developed infection control protocols to reduce the risk of coronavirus transmission, given the history of crisis management in the MERS and SARS epidemics, including avoiding nearest and direct contact with people with acute respiratory diseases, frequent hand washing right after direct contact with sick people or their environment, and avoiding unprotected contact with household and wild animals [8, 9].

### 1.3. The Problem

Social hypochondriasis is when people feel sick, but there is no reason to be sick. This phenomenon has been experienced in human societies for thousands of years, and it seems to be much more common than what is diagnosed in medicine. In a disease epidemic situation, people think they are sick when they see the first signs. This experience will vary depending on the type of illness, such as headache, dizziness, lethargy, shortness of breath, recurring coughs, chest pain, chills, and sore throats. When this happens, many people feel that they have symptoms. In many cases, one person is involved in the disease, and many other people consider themselves ill without real symptoms. In the corona epidemic, one of the main problems is the unseasonable visits to health centers. It caused both newly infected cases and weakened the ability to serve those in need. Unfortunately, the prevalence and transmission of COVID-19 are much higher than other similar viruses, and it lasts longer. Under critical circumstances, people get psychologically anxious by similar symptoms and visit medical centers. Therefore, a scientific method to detect infection by symptoms is useful to solve this problem.

### 1.4. Objective

Many investigators are analyzing and devising solutions for managing and screening COVID-19 disease in the real world. Given the research scale and the complexity of the issue, no commonly accepted criterion is provided for this context. In this paper, a GRC-based technique is presented to identify the presence or absence or severity of a disease from a person's symptoms.

The goal of this paper is to provide an algorithmic strategy for early detection or rejection of disease to avoid unnecessary congestion of people who are not infected in hospitals.

The proposed method acts as an intelligent prognosis for COVID-19 patients. However, it is not limited to COVID-19 and can be extended to other diseases. The smart system provided in this paper takes the information about the symptoms directly from the patient and screens whether they are sick or healthy according to the instructions and rules extracted. The paper is aimed at providing a reliable prognosis for patients to avoid attending medical centers as much as possible. The proposed approach can be developed as a web/mobile application to receive information directly from patients about symptoms without the need for chest X-ray and examinations. This performance is a great advantage, especially in epidemics of some diseases such as COVID-19.

The primary contribution of this paper is the following:

- We use granular computing early to diagnose the disease early; unlike the other approaches that utilize a narrow criterion, we simultaneously use all the rates of symptoms: that is, Fever, Headaches, dry cough, sore throat, shortness of breath, nausea, and vomiting
- The proposed solution is flexible so that new features can be added or subtracted. Also, the hierarchical nature and dynamics of this method have made it possible to consider all components
- The proposed algorithm is matchable. This means that by knowing and extracting rules from the training data, we do not need to reprocess the input variable
- Prompt diagnosis of the disease without the need for face-to-face visits vastly reduces the workload of medical centers

The paper is structured as follows: Section 2 supplies a summary of related work in granular computing, and Section 3 introduces and explores granular computations.  Section 4 defines the strategy, and finally, Section 6 presents the results and conclusions of this study.

## 2. Related Work

### 2.1. Granular

The concept of granular computing has been used in various fields such as artificial intelligence, clustering, machine learning, and databases [10, 11]. Therefore, it can be concluded that granular computing has been a hot research topic in recent years. The granules plays a key role in solutions to different issues with granular computing. If any classes, clusters, or groups are considered as granules, granular computing can be defined as a set of theories, methodologies, techniques, and tools that make use of granules to solve a problem [10, 12]. Yao introduced the information granulation concept, and he defined this concept in the field of fuzzy sets [10].

In 1999, Yao and Zhong [13] have shown that knowledge discovery and data mining are areas of computer science where granular computing can be used. If the granules are considered individually, the discovery of the relationships between them is the discovery of knowledge and data mining. These relationships can be unilateral or bilateral. The discovered relationships between the granular become the rules. If we look at the universe in terms of granulation, each granulation of the universe will have a different set of rules.

In granular computing, the steps of the fabrication, showing, and analysis of granules for problem-solving are the main components of the granulation process. It is necessary to establish a proper framework, to understand and investigate these issues. In 2002, Yao and Zhong and Yao, J.T. and Yao, Y.Y. [14, 15] introduce an information table as a notion and a model in the development of granular computing. In the proposed framework, with the assumption that the universe is not empty, each object has limited features. The universe can be divided into granular based on the values that these features have. This paper concludes that the proposed model, while simple, is very decisive in granular computing.

In 2004, Yao [10] focuses on the tasks of granulation and computing with granules. In an element of semantic and algorithmic, this paper analyses the construction, performance, and expression of granules, as well as directions and operations of computing and reasoning with granules. A division model of granular computing is also presented in this research. The model is based on the assumption that a finite set of the universe is granulated through a family of pairwise disjoint subsets. Finally, Yao infers that granular computing may be an essential principle that guides many problem-solving approaches.

Although granular computing in data mining and rule learning can be very beneficial, we did not find any beneficial research that utilizes granular computing in medical science. Because of the novelty of this computational model in data mining, all researchers in this field have introduced the model and proved its validity. In previous works, the predictive properties of this method are used in areas such as cloud computing [16, 17], geology [18], water science [19], and chemical [20, 21].

### 2.2. Artificial Intelligence

Due to the destructive effects of the coronavirus epidemic, computer science researchers have proposed techniques for detecting the disease in suspected individuals. Various solutions such as machine learning and deep learning are among these techniques. In this section, we will review these solutions.

In [22], the dataset including CT scans of 157 patients worldwide has been used as a training dataset. In this paper, an analysis is performed on images using an artificial intelligence method. To evaluate the results of the proposed solution, various datasets have been used and the presence or absence of disease has been investigated from CT scan images on them.

In [23], a dataset called COVIDx is made publicly; then, a combined human-machine design approach using the COVID_NET is presented. Using the COVIDx dataset simplifies the process of training and evaluating patient images. The dataset includes more than 1000 CT scan images of patients suspected of having COVID-19.

This paper focuses on three types of forecasting: (1) normal and without infection, (2) existence of infection that is not COVID-19, and (3) Coronavirus infection. A prototype is presented to show the results of these three types of predictions. Making these predictions will help the medical team make the correct decision to confirm the presence of COVID-19 disease or to treat other infections.

The solution presented in [24] is an approach for predicting the presence of COVID-19 disease in an infected person. This approach can predict the presence of COVID-19 disease six days before the first symptoms are presented. In this paper, the Integrated Moving Average Regression (ARIMA) is used as a model based on statistical analysis.

In [25], the machine learning approach is used to predict COVID-19 infection and to ask eight basic questions in the data. The data used consist of age, gender, and symptoms such as fever, cough, and headache. Out of a total history of 51831, 4769 positive patients were registered.

The main challenge in the proposed solutions is to predict the lack of required data as well as uncertainty; this has caused the accuracy of the proposed solutions to be very low. In the paper [26], a hybrid machine learning approach is proposed to increase the accuracy of prediction.

## 3. Granular Computing

Granular computing may be very useful in extracting knowledge and data mining. In granular computing, the granularization of the universe, the definition of granular, and the relationships between these granules are the main concepts. The values of the features of each object in the universe are shown in an information table [13]; each of these concepts is explained below:

*Granulation of a universe* means separating the universe into subsets or grouping particular objects into clusters. A granule, either fuzzy or crisp, may be viewed as a subset of the universe. A clan of granules containing every object in the universe is called a granulation, which provides a coarse-grained view of the universe. A granulation may consist of a family of either disjoint or overlapping granules. There are many granulations of the same universe [10].

*Description of granules* using a special logic language: the information presented in the information table can be deduced [16]. Along with an information table, a specific logic language can be defined to define an object or group of objects in the universe [14].

*Relationships between granules* in many situations: objects are usually grouped based on their relationships, such as in distinguished ability, similarity, proximity, or functionality [10].

The main idea of the granular computing model is how to solve a problem with various granulation methods. The term “granulation” refers to classifying each of the individual elements of the universe according to information about elements. The information table contains all the information about the objects in the universe. To build a granular tree, at the first stage, the universe is divided into partitions of the same class with a set of the atomic formula of attribute values. A rule can be expressed in the form, *φ*⟶Ψ where *φ* and Ψ are intensions of two concepts [27]. So the information table is one of the main concepts used in granular computing. The following section provides some details.

### 3.1. Information Table

An information table is used to display knowledge about the objects of the world. Each object has unique properties which are known by them and are described through the values of those properties in the data table. So two objects are equal if they have the same description [14, 15]. In a finite universe, all information about objects is presented by an information table in which objects are defined by their values on a finite set of attributes [13]. An information table is quadruple that is shown below [10, 13, 28].

(1) $$\begin{array}{c} S=\left\{U,\text{At},\left\{\text{Va}\;|\;a\in At\right\},\left\{I_{a}\;|\;a\epsilon At\right\}\right\}, \end{array}$$

where *U* is the universe, a finite nonempty set of objects, At is a finite nonempty set of attributes, Va is a nonempty set of values for *aϵ*At, and *I*_*a*_: *U*⟶Va is an information function.

In addition to granular computing, data mining and cluster analysis can also use the information table. As mentioned, the information in the information table is formatted through logical language [14]. In [29], the language of decision logic is introduced to describe an object or group of objects in the universe. An object is represented as a regular attribute-value pair. Similarly, a group of objects can be displayed. Formally, an atomic formula in the DL language is given by (*a*, *v*), where *aϵAt* and  *Vϵ*Va. If *φ* is a formula, the set *M*_*S*_(*φ*) is defined by

(2) $$\begin{array}{c} M_{S}\left(\varphi \right)=\left\{x\in U\right|\left.x\right|\left.=\varphi \right\}. \end{array}$$

*M*_*S*_(*φ*) is called the meaning of the formula *φ* in *S*. If *S* is understood, *M*_*S*_(*φ*) was written as  *M*(*φ*). A formula *φ* is said to be true in an information table *S*, written  *S*| = *φ*, if and only if  *M*(*φ*) = *U*; namely, *φ* is satisfied by all objects in the universe [13, 14, 30].

There is a fundamental problem in machine learning and data mining, and that is classification. There are two types of classification: supervised classification and unsupervised classification. In supervised classification, each object has a unique class-defined label that is predefined. Suppose an information table is used to describe a set of objects. Assume a unique attribute class taking class labels as its value. The set of attributes is expressed as  At = *F* ∪ {class}, where *F* is the set of attributes used to describe the objects. The goal is to find classification rules of the form *φ*⟶class = ci, where *φ* is a formula over *F* and ci is a class label [30].

## 4. The Proposed Method

In this paper, granular computing has been applied to solve a rule learning problem in data mining. From this perspective, basic granules are defined by an atomic formula and play a foundation role in the granular network. Pairs (*a* = *v*, *m* (*a* = *v*)) are a fundamental concept. Granule network construction is done by searching from top to bottom. In granular computing, one granule is defined by (attribute, value) at each step. In this approach, in a family of granules defined by values of an attribute, choosing a granule is more important than focusing on choosing the single partition at each stage [30]. The steps for building a granular network are described in Algorithm 1.

As mentioned earlier, granulation and the relationship between granules are essential issues in granular computing. To compute the size of a single granule, the relationship between two granules, and the relationship between a granule and a family of granules, some measurements are needed. Generality, confidence, coverage, and conditional entropy are four criteria for these goals and are done by the granule network algorithm. Each of them is explained in the following [27].

*Generality* for a single granular and a formula *φ*: generality is obtained by measuring the ratio *m*(*φ*) to the size of the universe, as shown below:

(3) $$\begin{array}{c} \text{Gen}\left(\varphi \right)=\frac{\left|m\left(\varphi \;\right)\right|}{\left|U\right|}. \end{array}$$

*Confidence* considers two formulas *φ* and  Ψ, the confidence of Ψ provided by *φ* is computed as follows:

(4) $$\begin{array}{c} \text{Conf}=\frac{\left|m\left(\varphi \text{ and }\Psi \right)\right|}{\left|m\left(\varphi \right)\right|}=\frac{\left|m\left(\varphi \cap \Psi \right)\right|}{\left|m\left(\varphi \right)\right|}. \end{array}$$

*Coverage* for two formulas *φ* and  Ψ: the coverage of Ψ provided by *φ* is computed as follows:

(5) $$\begin{array}{c} \text{Cov}=\frac{\left|m\left(\varphi \text{ and }\Psi \right)\right|}{\left|m\left(\Psi \right)\right|}=\frac{\left|m\left(\varphi \cap \Psi \right)\right|}{\left|m\left(\Psi \right)\right|}. \end{array}$$

*Conditional entropy*: this is a suitable technique for classification to make a decision tree [31]; this criterion is used for choosing attribute value. The conditional entropy is computed as follows:

(6) $$\begin{array}{c} \text{CEntropy}=-\overset{n}{\underset{\text{i}=1}{\sum }}\;p\left(\left.\Psi_{i}\right|\varphi \;\right)\log\;p\left(\left.\Psi_{i}\right|\varphi \right),\\ p\left(\Psi_{i}\;|\;\varphi \;\right)=\frac{\left|m\left(\varphi \cap \Psi_{i}\right)\right|}{\left|m\left(\varphi \right)\right|}. \end{array}$$

Note that entropy demonstrates the concept of inconsistency. For certain concepts, entropy reaches the minimum value, 0. This paper used a granular computing approach to extract rules for detecting novel COVID-19 diseases in humans according to observed symptoms.

To create the information table, we considered five classes numbered from one to five as below:

- Class 1: persons who have no symptoms of COVID-19
- Class 2: persons with slight symptoms who do not need a medical examination
- Class 3: persons who require an outpatient visit
- Class 4: persons who need hospitalization
- Class 5: persons who need special care

In this information table, each of the persons has been considered as an object which has some symptoms. These symptoms are regarded as attributes of these objects. Fever, headaches, dry cough, sore throat, shortness of breath, and nausea and vomiting are all symptoms that have been used in the attribute list. All these symptoms have been determined according to observed symptoms in patients. Each attribute has values in some fuzzy sets: low, medium, high, and very high.

The general model presented is shown in Figure 1. In this model, it is assumed that a person who has some related symptoms uses the application and, depending on the level of symptoms, selects one of the very low, low, medium, high, or very high options. The details of this process are shown in Figure 1.

## 5. Proposed

In this study, the mechanical inference of classification rules for COVID-19 classification using a GRC algorithm applies to apply concepts, such as generality, confidence, coverage, and entropy (already defined), in seven essential steps. Algorithm 2 shows the steps.

### 5.1. Example

Here, we show an exemplary example showing how the proposed algorithm works and computes the statistical parameters because our algorithm is supplied for rule extraction of static data. Its execution is also clear in the small dataset. Consider the dataset in Table 1.

This information table using all data available online at the Worldometer International Team's website has been built.

In the second stage, some formulas have been defined to be able to granulate the universe. These formulas are listed in Table 2.

In the next step, the algorithm calculates coverage, confidence, and entropy for all formulas provided in the previous stage for each class. To produce a COVID-19 detection classification with minimum uncertainty, a subset of an attribute value with high coverage, confidence, and lowest entropy must be found. At this stage, it is important that redundancy is inevitable and must be taken into account.  Figure 2 shows the general overview of the steps performed in the presented method.

In this example, a dataset consisting of 20 patients with COVID-19 symptoms was selected from the report on the Worldometer International Team's website [32]. All data have been classified by experts in five classes. After the execution of the granular algorithm, the final tree was constructed.  Figure 3 shows the result. By executing the algorithm on this training data, eight rules are inferred at three levels. The partnership of inactive granules at three levels covers the universe set. Each node of the granule decision tree is marked by a value of the attribute, and each branch is marked with a value of the parent attribute. The results of accuracy are computed by

(7) $$\begin{array}{c} \frac{k}{k+n}. \end{array}$$

The number of objects that are correctly classified by a rule is indicated by *k*. In other words, the objects are correctly placed in their respective classes. *n* also shows the number of objects that are classified not correctly. To provide a simulation-based assessment, it is essential to consider all the paths of a complete system. All data used in this study were retrieved from the website of the Ministry of Health.

The dataset was downloaded, translated into English, and can be accessed at https://github.com/nshomron/covidpred.

The training and experimental set used contains the signs of 51831 people tested, on March 22-31 and April 1-7, 2020, respectively.

We evaluated the effectiveness of GRC using AMD PC with a 3.2 GHz CPU and 8 GB memory, running Microsoft Windows 8 Professional and Matlab R2021b.

The proposed granular computing algorithm was performed on the symptoms of COVID-19 patients, and finally, some of the rules derived from it are shown below:

1. **IF** shortness of breath is medium, **THEN** the person requires an outpatient visit
2. **IF** nausea and vomiting is low **AND** fever is high, **THEN** the persons need hospitalization
3. **IF** nausea and vomiting is low **AND** fever is medium **AND** dry cough is low, **THEN** the persons have no symptoms of COVID-19
4. **IF** nausea and vomiting is low **AND** fever is very high **AND** dry cough is medium, **THEN** the persons need special care

Determining the vulnerability of the disease is a multicriterion decision class that is always associated with uncertainties due to its dependence on parameters and expert opinion. Each of the multicriterion decision-making methods manages certain aspects of luck, and none of them can manage uncertainty comprehensively. Using a granular computation model is a suitable method for extracting rules with zero incompatibility to manage uncertainty in this research which has been proposed and implemented. In this model, the rules were removed from the sample data with zero incompatibility. In this model, rules are formed, compared, and extracted in attribute pairs, not based on single attributes.

Using the general similarity relationship in the formation of the granular computation model, considering the overlapping boundaries, the limitation of definite limits is also removed. Also, more rules can be extracted using this model. In this method, due to the overlapping of the boundaries, the values of their attributes are placed at the limits, and they are classified by more than one rule, which in turn increases the accuracy of the final output.

In this section, we have compared the proposed approach with two other approaches qualitatively [33, 34]; in this comparison, fast and in-time detection has been the aim of all three approaches.  Table 3 summarizes the comparison results. In this table, it is clear that the proposed method has been able to operate faster than the other two methods without the need for face-to-face examination.

The results of the classification based on the granular computing model show that 5% of the studied population have no symptoms of the disease, 22% have mild symptoms that do not need a medical examination, 18% of them require an outpatient visit, 30% need hospitalization, 14% need intensive care, and only a few cases are not classified by this method. In this paper, only a few apparent symptoms are considered.  Figure 4 shows the COVID-19 vulnerability degree in the proposed method.

## 6. Conclusion

Due to the epidemic of COVID-19 disease and the lack of a suitable tool for learning and detecting illness according to symptoms, this paper presents an algorithm that uses granular computing to determine the presence or absence of even illness severity. The proposed research shows an application of granular computing in medicine. At this time and in the global epidemic of an unknown coronavirus, it can be a practical step in providing medical assistance. By considering more features such as the patient's age, gender, or even the genome, the proposed method can improve detection accuracy. In this paper, we tried to discuss the nature of the granular approach for use in medicine and to help develop computer applications in this field.

In this paper, we wanted to demonstrate that experience has shown that granular computing, in which a model of information is processing, can be helpful in various fields, explore relationships between data, and extract meaningful information for us.

Association rules are one of the available methods to find hidden knowledge about the universe. Without enough information about the universe, the objects in it are not identified. To obtain a description of these in a universe of which we have insufficient information and to derive the laws governing it, the objects of the universe are classified based on an indistinguishable relation. This classification forms the granules. The granules are processed by granular computing, and possible patterns and rules are extracted.

According to the scopes noted in the study, issues for additional study and research are suggested:

- Provide a standard method for accurately determining the characteristics

Determining the specificity of each problem is one of the most critical phases of problem-solving. The specifications involved in the calculations must be selected correctly.

(ii) Use of the lie detection algorithm before creating the information table to consider false information

Since this method is a human-centered solution, there is a need to reduce human error with intelligent algorithms.

(iii) Check and improve the execution time of the algorithm by increasing or decreasing the amount and complexity

In future work, the execution time and complexity of this method can be discussed.

(iv) Collect up-to-date and comprehensive data and evaluate the proposed solution using them

To assess the proposed solution, we need actual data and its labeling by an expert.

## Figures and Tables

**Figure 1:** Deployed proposed granular model for assessing and detecting COVID-19 in clinical application.

**Figure 2:** Steps performed in the proposed method.

**Figure 3:** Granular tree of the proposed method.

**Figure 4:** Vulnerability degree in the proposed method

**Algorithm 1:** Granular network construction algorithm [30].

**Algorithm 2:** Algorithm to construct granular tree.

**Table 1:** Information table for COVID-19 patient (L: low; M: medium; H: high; VH: very high).

Object	Fever	Headaches	Dry cough	Sore throat	Shortness of breath	Nausea and vomiting	Class
1	L	M	L	M	M	M	3
2	VH	L	H	H	L	L	4
3	VH	L	M	H	H	L	5
4	H	L	VH	H	L	L	4
5	M	VH	VH	H	L	L	2
6	VH	L	M	H	L	L	4
7	L	VH	L	H	M	L	3
8	L	VH	L	M	VH	M	4
9	VH	H	H	M	VH	M	4
10	M	H	H	M	L	L	2
11	L	M	L	M	M	M	3
12	VH	L	H	H	H	L	4
13	M	L	VH	H	H	L	5
14	H	L	H	H	L	L	4
15	M	H	H	H	L	L	2
16	M	H	H	L	L	L	2
17	L	M	L	H	M	M	3
18	M	M	L	L	L	L	1
19	VH	M	M	M	L	L	5
20	M	H	L	M	L	L	2

**Table 2:** All formulas according to information table and fuzzy sets of attributes (L: low; M: medium; H: high; VH: very high).

Fever (F)	Headaches (H)	Dry cough(DC)	Sore throat (ST)	Shortness of breath(SB)	Nausea and vomiting (NV)
F = L	H = L	DC = L	ST = L	SB = L	NV = L
F = M F = H F = VH	H = M H = H H = VH	DC = M DC = H DC = VH	ST = M ST = H	SB = M SB = VH	NV = M

**Table 3:** Qualitatively comparison two approaches with the proposed approach.

Reference	Method	No in-person visits	No need to X-ray	No need to CT-scan	Aim	Accuracy
[32]	HDNN	×	×	×	Fast detection	99%
[33]	DL with RF	×	×	✓	Fast detection	97.29%
Proposed	GRC detection	✓	✓	✓	Fast detection	89%

## Data Availability

The dataset was downloaded, translated into English, and can be accessed at https://github.com/nshomron/covidpred.
